# Adoption and Safety Evaluation of Comfortable Nursing by Mobile Internet of Things in Pediatric Outpatient Sedation

**DOI:** 10.1155/2022/3257101

**Published:** 2022-06-25

**Authors:** Qiuying Xiao, Bingqing Wu, Wei Wu, Rui Wang

**Affiliations:** ^1^Comfort Medical Management Center, Hunan Children's Hospital, Changsha 410011, China; ^2^Department of Anesthesia Surgery, Hunan Children's Hospital, Changsha 410011, China

## Abstract

The aim of study was to explore the application effect and safety of comfortable nursing based on optimized mobile Internet of Things (MIoT) in the clinical sedation and diagnosis of mycoplasma pneumoniae pneumonia (MPP) in children. A total of 70 children with MPP admitted to the respiratory clinic of hospital were randomly selected and divided into a control group (comfortable nursing mode) and an observation group (comfortable nursing mode based on optimized MIoT), with 35 cases in each. The nursing effects and safety were compared between groups. The results showed that the node jitter rate, delivery success rate, and congestion times of the multilayered sensing algorithm were better than those of the mobile relay area segmentation algorithm and the wedge merge-energy hole elimination area segmentation algorithm. The CD-RISC resilience score of the observation group ((94.72 ± 1.58) points), the proportion of children with Frankl-3 and 4 points (90%), and the comfort level ((95.01 ± 5.68) points) were higher than those of the control group ((64.12 ± 1.62) points, (33.33%), and (55.23 ± 6.18) points) (*P* < 0.05). After treatment, the proportion of children with HRCT image lesions in the observation group was lower than that in the control group (*P* < 0.05). After treatment, the FEV1 ((85.71 ± 5.23) % vs. (68.26 ± 5.90) %) and FEV1/FVC ((74.22 ± 2.12) % vs (64.38 ± 2.34) %) of the observation group were significantly better than those of the control group (*P* < 0.05). The results showed that the incidence of adverse reactions in the observation group (14%) was significantly lower than that in the control group (46%) (*P* < 0.05). MIoT-assisted comfort nursing based on multilayer perception region segmentation algorithm can more effectively relieve the emotions of children in MPP outpatient department during sedation and diagnosis and treatment, improve the therapeutic effect and safety, and is worthy of clinical promotion.

## 1. Introduction

With the rapid development of social science and technology, various diagnosis and treatment technologies in the medical industry have made great progress. Therefore, the traditional medical model of the medical industry has also undergone great changes. It is found that the traditional biomedical model has been transformed into a new social-psychological-biomedical model [1, 2]. In other words, modern medical treatment pays more attention to the influence of patients' psychological factors on the occurrence, development, treatment, and prognosis of various diseases, such as depression caused by maternal anxiety and tension [3] and the tension of patients before surgical anesthesia [4]. Comfortable nursing is a new professional nursing mode in clinic. It was proposed by Kolcaba and has the advantages of high integrity, strong pertinence, and good effect [5, 6]. At present, comfortable nursing has been widely used in all aspects of clinical diseases, with increasing the comfort of patients as the main work content. Studies have shown that comfort care can alleviate patients' abnormal emotions (such as tension, fear, and anxiety) [7]. As the incidence of children's lung infection diseases gradually increases, comfortable nursing has been widely applied in the outpatient diagnosis and treatment of children's lung diseases, especially pulmonary infectious diseases [8]. Pulmonary infection is a disease with a very high clinical incidence, and the onset is more acute. In severe cases, a large amount of mucus will be secreted to block the airway. If timely treatment and care cannot be given, it will bring certain life risks to patients, among which mycoplasma pneumoniae (MP) infection is more common [9]. Mycoplasma pneumoniae pneumonia (MPP) accounts for a high proportion of all pneumonia, and its clinical manifestations are diverse, resulting in varying degrees of lung function impairment. Therefore, timely and accurate diagnosis and treatment are required [10]. Since some pulmonary examination methods (such as pulmonary bronchoscope) may cause discomfort to patients, sedation (anesthesia) is also necessary in the pulmonary clinic. In addition, chest HRCT and lung function detection are also common methods of lung disease examination, which are of good clinical adoption value.

In addition, the sharp increase of clinical patients poses a great challenge to the work level and intensity of nursing staff, resulting in the impact on the service quality of the medical industry. Therefore, how to reasonably allocate medical resources and improve the level of medical services has become a key issue of concern [11]. The emergence of Internet of Things technology (information carrier of network interconnection based on Internet and telecommunication network) undoubtedly provides technical conditions, and this technology has been widely applied in the medical field [12]. Mobile Internet of Things (MIoT) [13] is the integration of mobile communication technology and traditional Internet of Things technology, which plays an important role in hospital information management. MIoT has the characteristics of fast information transmission, low location restriction, and low management cost, so that medical institutions can provide more convenient and better services [14]. However, some studies have proposed that MIoT nodes are prone to frequency interruption when topology changes frequently [15]. Therefore, it is necessary to segment and strengthen the network sensing area to improve the stability of the network. Someone pointed out a MIoT region segmentation algorithm based on multilayered perception. The research results show that the algorithm can better improve the stability of the network and improve the data transmission [16]. At present, this technology has been well adopted in medical informatization and mobile nursing.

In summary, the application effect and safety of comfortable nursing based on optimized MIoT in outpatient sedation of children MPP were studied. It was hoped that more effective care methods can be provided for children with respiratory diseases to improve the treatment effect and prognosis of patients.

## 2. Research Methods

### 2.1. Subjects

In this study, 70 children with MPP admitted to the hospital from September 2020 to September 2021 were randomly selected as the research objects. There were 40 males and 30 females, ranging in age from 4 to 12 years old, with an average age of (6.24 ± 1.70) years old. Random number table method was used to divide the children into control group and observation group. Patients in the control group were sedated with comfortable nursing mode. Patients in the observation group were treated with sedation nursing based on the comfort nursing mode of optimized MIoT. The number of children in both groups was 35. Then, the effect and safety of outpatient sedation nursing in the two groups were evaluated combined with CT examination and lung function examination. This study had been approved by ethics committee of hospital, and the patients and their families signed the informed consent form.

Inclusion criteria: (i) children who had bad mood before MPP examination and needed sedation nursing; (ii) the age range of all the children was 4 years and above; (iii) children with MPP had normal mental state and consciousness; (iv) all the children and their families agreed to undergo CT and lung function examination.

Exclusion criteria: (i) children who refused to cooperate with examination and treatment during the study; (ii) children with MPP who cannot receive complete treatment evaluation; (iii) children complicated with other respiratory diseases.

### 2.2. MIoT Region Segmentation Algorithm

MIoT node has the characteristics of movement and fast topology change, which leads to the unknowability of the transmission direction of the node. The previous processing methods diversify the cluster head nodes, but cannot make full use of the information of each node. Therefore, it is necessary to further standardize the information that complete the node feature extraction, so as to better segment the network area. That is, multilayered perception segmentation of network structure is adopted.

The structure of the Internet of Things is generally divided into three categories: sensor network, transmission network, and application network (Figure 1). Sensor network—the main function is monitoring; transmission network—the main function is to transmit information to external Internet (such as Internet, radio, and television network, NGN); application network—edit information.

It is assumed that the space of topological nodes in the whole network is *Q*, and any node in the mobile network structure in this space is *w*, when the state of *w* is in motion mode, the total number of nodes within the radius of the node can be expressed as *e*. According to the above, it is supposed that the interaction matrix of the target data at this time is *R*, and there is the following expression.

(1) $$\begin{array}{c} R=\left\{\begin{array}{c} T\left(w,1\right),\\ T\left(w,2\right),\\ \vdots ,\\ T\left(w,e\right). \end{array}\right. \end{array}$$

*T*(*w*, *e*) represents the interaction vector of the target data. When the data exchange between *w* and *e* does not exist, the various elements in *R* are 0. *w* is set as the cluster head node, the *T*(*w*, *e*) value plus 1 when the data within its range is exchanged. In other words, the higher the *T*(*w*, *e*), the closer the relationship between *w* and *e*. Based on the above conclusion, it is necessary to initialize all nodes in the network in order to extract enough *w*. In order to keep the network smooth, it adopts the multilayered perception algorithm composed of network layer, transmission layer, and final aggregation layer.

If the number of *w* is *n*, the element state vectors *Un* and *On* in network layer and transmission layer need to satisfy the following equation.

(2) $$\begin{array}{c} Un=\left\{\begin{array}{c} T\left(w,1\right),\\ T\left(w,2\right),\\ \vdots ,\\ T\left(w,e\right), \end{array}\right. \end{array}$$

(3) $$\begin{array}{c} On=\left\{\begin{array}{c} O\left(w,1\right),\\ O\left(w,2\right),\\ \vdots ,\\ O\left(w,e^{\prime }\right). \end{array}\right. \end{array}$$

*T*(*w*, *e*) represents the interaction vector between *w* and the *e* node; *O*(*n*, *e*′) indicates the interaction vector between *w* and the *e* cluster head node. In order to improve the efficiency of solution, Equations (2) and (3) are improved.

(4) $$\begin{array}{c} P\in \left[\begin{array}{c} Un=1\\ On\cap Q \end{array}\right.=\frac{1}{1+z^{-\left(kn+\int_{j=1}^{m}SnjD\left(n,m\right)\right)}}, \end{array}$$

(5) $$\begin{array}{c} P\in \left[\begin{array}{c} On=1\\ Un\cap Q \end{array}\right.=\frac{1}{1+z^{-\left(gn+\int_{j=1}^{v}SnjD\left(n,v\right)\right)}}. \end{array}$$

*s* represents the exchange weight of *kn* (cluster head node in the segmentation region) and *gn* (cluster head node queried). After a series of calculations, the state vector *G* in the final output layer can determine that the network is in a stable state.

(6) $$\begin{array}{c} Gn=\left\{\begin{array}{c} g^{n1},\\ g^{n2},\\ \vdots ,\\ g^{nm}. \end{array}\right. \end{array}$$

When Equations (4) and (5) are stable, the state vector in the final output layer is *G*, and further vector analysis is carried out. The region segmentation algorithm based on the opportunistic collision information extraction mechanism is used. It is assumed that there are *m* components that are not 0, and Equation (7) can be obtained.

(7) $$\begin{array}{c} \bar{Gn}=\left\{\begin{array}{c} g^{n1},\\ g^{n2},\\ \vdots ,\\ g^{nm}. \end{array}\right. \end{array}$$

*g* ^*nm*^ represents the component corresponding to *m* components that are not 0; $\bar{Gn}$ means the region segmentation vector obtained by reordering *g*^*nm*^. Then, the Lagrange function is used to optimize the opportunity collision information extraction process, and the following equation can be obtained.

(8) $$\begin{array}{c} L=\max\int_{n=1}^{S}\int_{l=i}^{m}H_{nl}^{\omega_{nl}}\left[g_{nk}-g_{nm}\right]. \end{array}$$

*L* represents the objective function, *S* represents the number of ordinary nodes, *H*_*nl*_ denotes the chance collision degree between ordinary node *n* and cluster head node *gn*, and *ω*_*nl*_ represents the redundancy factor.

(9) $$\begin{array}{c} \int_{n=1}^{S}H_{nl}<0, \end{array}$$

(10) $$\begin{array}{c} \int_{l=i}^{m}H_{nl}=1, \end{array}$$

(11) $$\begin{array}{c} 0\leq H_{nl}\leq 1. \end{array}$$

Through the above contents, the opportunity collision degrees *H*_*nl*_ and *g*^*nm*^ can be obtained.

NS2 simulation environment was used to verify the performance of the algorithm. The network parameters were set as follows: node density ≥ 5•100 m^−2^, moving speed ≤ 30 m•s^−1^, deployment area 1,024 × 1,024 m^2^, 5 G network, regional clustering mobile model, segmentation number ≥ 5, and running time ≤ 50 min. The performance of the algorithm was evaluated by node jitter rate, congestion times, and data delivery success rate.

### 2.3. Comfortable Nursing Method

Comfortable nursing—adopted comfortable nursing performed intervention from the treatment environment, medical staff, and treatment process (before treatment, during treatment, and after treatment). The treatment environment was quiet to make children feel warm and comfortable; medical staff needed a gentle expression; appropriate rewards could be given according to the performance of children during treatment. Before diagnosis and treatment, children must be familiar with the environment of the examination room and interested. In the diagnosis and treatment process, targeted diagnosis and treatment were adopted, such as cooling and warm care for fever and chills. Oxygen inhalation was performed for hypoxemia children. At the same time, the computer played soft and relaxing music, and language encouragement was given, so that the children relaxed. After the diagnosis and treatment, children were given praise and some small gifts, and pulmonary care education was performed during treatment. In this study, MIoT was used to provide real-time understanding of the situation of children and formulate reasonable nursing, treatment, education, and follow-up, thus improving the treatment effect of children and reducing the recurrence rate of children.

### 2.4. CT Examination Method

High-resolution CT (HRCT) scanning of lung was performed by high resolution CT. Range was from apex of lung to diaphragm. Parameters were tube voltage of 120 kV and layer thickness of 1.5 mm. The lung characteristics of HRCT were observed, including increased lung texture, rope shadow, ground glass shadow, small patchy shadow, large patchy consolidation, atelectasis, bronchiectasis, pleural effusion, and hilar mediastinal lymph node enlargement.

### 2.5. Pulmonary Function Test

Lung function examination was performed using lung function instrument. Before checking, calibrate environmental parameters and capacity were adjusted and standardized. The estimated value can be automatically generated according to age, height, and weight parameters. The position was standing with head natural, inhaling deeply to total lung capacity (TLC), and exhaling to functional residual capacity (FRC). The time-volume curve and flow-volume curve were plotted, and the average value of the three best test values was deemed as the judgment result. One second forced expiratory volume (FEV1) and FEV1/forced vital capacity (FVC) (FEV1/FVC) were observed.

### 2.6. Observation Indicators

The psychological resilience of the children in the control group and the observation group before treatment was compared (assessed by the Connor-Davidson Resilience Scale (CD-RISC) (Table 1)). The degree of cooperation in the treatment process was assessed by the Frankl scale (Table 2). Posttreatment comfort (level of comfort) was assessed by the General Comfort Questionnaire (GCQ) (Table 3).

The HRCT and pulmonary function test results before and after three months of treatment, and the incidence of adverse reactions (including abnormal nervous system, nausea and vomiting, and abnormal skin reactions) after treatment was compared between the two groups.

### 2.7. Statistical Methods

The results were statistically analyzed by SPSS 22.0 statistical software. The measurement data were expressed as mean ± standard deviation($\overset{®}{x}$ ± *s*). The independent sample *t*-test was used. The enumeration data were expressed as the number of cases or percentage. *χ*^2^ test was used. The difference was statistically significant when *P* < 0.05.

## 3. Results

### 3.1. Performance Analysis of the Algorithm

The proposed algorithm was compared with the moving relay region segmentation algorithm [17] and the wedge merge-energy cavity elimination region segmentation algorithm [18]. The results were shown in Figure 2. It was found that when the network running time was 50 min, the node jitter rate (0.1%) of this algorithm was significantly lower than that of the other two algorithms (30.09% and 69.89%), and the data delivery success rate (89.97%) was higher than that of the other two algorithms (71.08% and 53.34%); when the node density was 55•100 m^−2^, the number of network data congestion times (302 times) of this algorithm was lower than that of the other two algorithms (554 times and 769 times).

### 3.2. Comparison of General Data

The general data (gender, age, body weight, etc.) of the children were compared. The results showed that there was no significant difference in gender distribution, age distribution, and body weight distribution between the two groups (*P* > 0.05), suggesting that the comparison between the groups had certain feasibility (Figure 3).

### 3.3. Comparison of Score Results

The conditions of the control group and the observation group before, during, and after treatment were statistically compared. The results were as follows: before treatment, the average CD-RISC total psychological flexibility score of the observation group ((94.72 ± 1.58) points) was higher than that of the control group ((64.12 ± 1.62) points) (*P* < 0.05); during treatment, the Frankl score of the observation group was 3 and 4 points in 27 cases (90%), and the Frankl score of the control group was 3 and 4 points in 10 cases (33.33%), *P* < 0.05. After treatment, the comfort score of the control group ((55.23 ± 6.18) points) was significantly lower than that of the observation group ((95.01 ± 5.68) points) (*P* < 0.05) (Figure 4).

### 3.4. HRCT Examination Results

Figure 5 showed the comparison of the HRCT examination results of the two groups of children before treatment and after three months of treatment. HRCT images of the two groups of children before treatment showed increased lung markings, streak shadows, ground glass shadows, small patchy shadows, large consolidation shadows, atelectasis, bronchiectasis, pleural effusion, and hilum mediastinal lymphadenopathy. There was no significant difference in the proportion of the number of children (*P* > 0.05). After treatment, the above HRCT manifestations of the two groups of children were significantly reduced compared with those before treatment. In the observation group, the proportion of children with lung markings increased (11% vs. 29%), streak shadows (3% vs. 9%), ground glass shadows (6% vs. 17%), small patchy shadows (9% vs. 17%), large patchy consolidation (11% vs. 29%), atelectasis (14% vs. 29%), bronchiectasis (9% vs. 14%), pleural effusion (0 vs. 6%), and hilar and mediastinal lymphadenopathy (0 vs 9%) was lower than that in the control group (*P* < 0.05).  Figure 6 showed HRCT images of the two groups of children before and after treatment, which showed that the lung symptoms of the children were significantly improved.

### 3.5. Pulmonary Function Test Results

Figure 7 showed the mean values of FEV1 and FEV1/FVC in pulmonary function tests of the two groups of children before and after treatment. Before treatment, the FEV1 was ((49.12 ± 5.89) % vs. (50.34 ± 5.51) %) and FEV1/FVC was ((50.33 ± 1.76) % vs. (50.55 ± 1.87) %) in the observation group and the control group. There was no significant difference in the mean values of FEV1 and FEV1/FVC between the two groups before treatment (*P* > 0.05). After treatment, the FEV1 ((85.71 ± 5.23) % vs. (68.26 ± 5.90) %) and FEV1/FVC ((74.22 ± 2.12) % vs. (64.38 ± 2.34) %) of the observation group and the control group were significantly improved compared with those before treatment, and the FEV1 and FEV1/FVC of the observation group were significantly better than those of the control group (*P* < 0.05).

### 3.6. The Incidence of Adverse Reactions

According to statistics in Figure 8, there were 3 cases of neurological abnormalities, 6 cases of nausea and vomiting, and 7 cases of abnormal skin reactions in the control group after treatment, with a total incidence rate of 46%. In the observation group, there were 1 case of neurological abnormalities, 2 cases of nausea and vomiting, and 2 cases of abnormal skin reactions after treatment, with a total incidence rate of 14%. After comparison, the incidence of adverse reactions in the observation group was significantly lower than that in the control group (*P* < 0.05).

## 4. Discussion

Comfort care model, as a new type of medical care, has played an important role in various clinical diseases, such as postpartum care of parturients [19], care of patients with advanced cancer [20], and perioperative care of various diseases [21, 22]. Among them, respiratory department diagnosis and treatment is particularly important for comfort care models due to the wide range of populations faced, especially for children. It is increased pressure on the medical industry to diagnose and treat due to the unlimited age of patients. The MIoT has helped the medical industry alleviate this problem to some extent to achieve the efficiency and accuracy of nursing work and improve the quality of clinical care. MIoT can make patients and medical staff communicate without time limit and place limit, so that medical staff can timely understand the patient's condition and develop effective diagnosis and treatment plan and postoperative education.

In this study, the sedation assistance effect of MIoT in comfortable nursing mode was explored with the children treated by MPP in outpatient department as the research object. The results showed that the average CD-RISC total psychological flexibility score (94.72 ± 1.58 points), proportion of children with Frankl score of 3 and 4 points (90%), and comfort level (95.01 ± 5.68 points) in the observation group were higher than those in the control group (64.12 ± 1.62 points, 33.33% points, and 55.23 ± 6.18 points) (*P* < 0.05). The results suggested that the real-time understanding of children's personality and emotions through MIoT medical information system to develop targeted sedation and nursing programs can effectively alleviate the adverse emotions and resistance during the treatment of children. Kelly et al. (2020) [23] pointed out that the Internet of Things can simplify and strengthen the provision of medical services, actively predict the health problems of patients, and facilitate the diagnosis, treatment, and monitoring of patients inside and outside the hospital. By comparing the HRCT and pulmonary function test results of the two groups of patients before and after treatment, it was concluded that, in the observation group after treatment, the proportion of children with manifestations of increased lung markings (11% vs. 29%), streak shadows (3% vs. 9%), ground glass shadows (6% vs. 17%), small patchy shadows (9% vs. 17%), massive consolidation (11% vs. 29%), atelectasis (14% vs. 29%), bronchiectasis (9% vs. 14%), pleural effusion (0 vs. 6%), and hilar and mediastinal lymphadenopathy (0 vs. 9%) was lower than that of the control group (*P* < 0.05). After treatment, the FEV1 ((85.71 ± 5.23) % vs. (68.26 ± 5.90) %) and FEV1/FVC ((74.22 ± 2.12) % vs. (64.38 ± 2.34) %) of the observation group were significantly better than those of the control group (*P* < 0.05). The results suggested that the real-time monitoring of the conditions of patients inside and outside the hospital through MIoT can improve the treatment of children. Liu et al. (2022) [24] combined MIoT technology and nursing information management system for the treatment, nursing, and rehabilitation guidance of cervical spondylosis, which improved the quality of nursing services, improved work efficiency, and improved the patient's condition. In terms of safety assessment during the nursing process, the incidence of adverse reactions in the observation group (14%) was significantly lower than that in the control group (46%) (*P* < 0.05). The above results suggested that in the case of effective sedation nursing for children, understanding the condition of children and giving corresponding treatment and nursing methods can effectively reduce the incidence of risk events caused by conflict in children, with high safety. This is consistent with the findings of Lakhan et al. (2021) [25].

Because MIoT is prone to frequency interruption in the process of data transmission, it uses multilayered perception network sensing area segmentation algorithm to optimize MIoT, so that its transmission process is more stable. The results show that the node jitter rate and the success rate of data delivery in this algorithm are superior to those in the mobile relay region segmentation algorithm and the wedge merge-energy cavity elimination region segmentation algorithm under the same operation time; when the node density is the same, the number of network data congestion (302 times) is lower than that in the other two algorithms (554 times and 769 times), suggesting that the algorithm has better network region segmentation effect and stronger data congestion control ability. This is consistent with the findings of Liao et al. (2020) [26] and Shi and Suo (2020) [27], suggesting that the results have some accuracy.

## 5. Conclusion

In this study, MIoT-assisted comfort nursing based on multilayer perception region segmentation algorithm was used to carry out sedation nursing diagnosis and treatment for children with MPP in outpatient department, and its application effect and safety were analyzed through pulmonary function examination and the occurrence of adverse reactions. The results showed that MIoT-assisted comfort nursing based on multilayer perception region segmentation algorithm can more effectively relieve the emotions of children in MPP outpatient department during sedation and diagnosis, improve the therapeutic effect and safety, and is worthy of clinical promotion. However, this study only took MPP children as the research object, the coverage of the disease is not comprehensive enough, and further research is needed. However, only children in the department of stomatology were studied, and the disease coverage was not comprehensive enough, which still needs further exploration. The results showed that the auxiliary role of MIoT technology in medical information system can be affirmed to a certain extent, revealing the good application prospect of MIoT technology in clinical practice.

## Figures and Tables

**Figure 1:** Structure of Internet of Things.

**Figure 2:** Performance comparison of algorithms. (a) Multilayered perception segmentation. (b) Moving relay. (c) Wedge merge—energy cavity elimination.

**Figure 3:** Comparison of basic information of patients.

**Figure 4:** Comparison of evaluation results between control group and observation group. ∗Compared with the control group, *P* < 0.05.

**Figure 5:** Comparison of HRCT examination results. (a) Increased lung markings. (b) Streak shadows. (c) Ground glass shadows. (d) Small patchy shadows. (e) Large consolidation shadows. (f) Atelectasis. (g) Bronchiectasis. (h) Pleural effusion. (i) Lung portal mediastinal lymphadenopathy. ∗Compared with the control group, *P* < 0.05.

**Figure 6:** HRCT images before and after treatment.

**Figure 7:** Pulmonary function test results. ∗Compared with the control group, *P* < 0.05.

**Figure 8:** Incidence of adverse reactions. ∗Compared with the control group, *P* < 0.05.

**Table 1:** CD-RISC scoring scale.

Dimension	Toughness	Strength	Optimism
Score (points)	0 ~ 52	0 ~ 32	0 ~ 16

∗Positive correlation between resilience and CD-RISC points.

**Table 2:** Frankl scoring scale.

Score (points)	1	2	3	4
Performance	Refusal, pain	Uncooperative, reluctant	Adaptative, indifferent	Active cooperation

∗Positive correlation between patient compliance and Frankl scale score.

**Table 3:** Kolcaba comfort scale.

Dimension	Environment	Physiology	Social culture	Mentality
Score (points)	0 ~ 12	0 ~ 32	0 ~ 16	0 ~ 52

∗Positive correlation between patient comfort and Kolcaba comfort scale score.

## Data Availability

The data used to support the findings of this study are available from the corresponding author upon request.
